RETRACTED

# Nitroxyl (HNO): A Reduced Form of Nitric Oxide with Distinct Chemical, Pharmacological, and Therapeutic Properties

**DOI:** 10.1155/2016/4867124

**Published:** 2015-12-07

**Authors:** Mai E. Shoman, Omar M. Aly

**Affiliations:** Department of Medicinal Chemistry, Faculty of Pharmacy, Minia University, Minia 61519, Egypt

## Abstract

Nitroxyl (HNO), the one-electron reduced form of nitric oxide (NO), shows a distinct chemical and biological profile from that of NO. HNO is currently being viewed as a vasodilator and positive inotropic agent that can be used as a potential treatment for heart failure. The ability of HNO to react with thiols and thiol containing proteins is largely used to explain the possible biological actions of HNO. Herein, we summarize different aspects related to HNO including HNO donors, chemistry, biology, and methods used for its detection.

## 1. Nitric Oxide (NO)

Biological activities associated with nitrogen oxide species are the subject of intense and current research interest. Much of this interest stems from the discovery of endogenous NO generation [1], a significant event that represents a fundamentally new paradigm in mammalian cell signaling. Prior to this finding, the idea that a small, freely diffusible, reactive molecule (known more for its toxicity) could be biosynthesized in a highly regulated fashion and elicit specific biological functions was unheard of and, for some at the time, heretical [2]. Most attention has been focused on NO since it is generated directly in mammalian cells by a family of enzymes referred to as the NO synthases (NOS) which converts the terminal guanidino nitrogen of l-arginine into NO (Scheme 1) [3, 4].

NO was described more than 30 years ago as a ligand of the NO-sensitive soluble guanylate cyclase (NO-sensitive sGC), the enzyme that catalyzes the conversion of guanosine 5′-triphosphate to guanosine 3′,5′-cyclic monophosphate (cGMP) [5]. NO activation of sGC involves coordination to a regulatory ferrous heme on the protein resulting in an increase in catalysis and a subsequent increase in intracellular cGMP [2]. Increased levels of cGMP within vascular smooth muscle result in vasodilatation [5]; thus continual release of NO regulates vascular tone and assists in the control of blood pressure [6]. In addition, NO increases the level of cGMP in platelets, and this is thought to be the mechanism by which it inhibits platelet function [7]. In the vasculature, NO also prevents neutrophil/platelet adhesion to endothelial cells, inhibits smooth muscle cell proliferation and migration, regulates programmed cell death (apoptosis), and maintains endothelial cell barrier function [8].

Along with NO, significant interest also exists for its oxidized congeners nitrogen dioxide (NO_2_), peroxynitrite (ONOO^−^), and nitrite (NO_2_^−^), among others. This attention may be a function of the facility by which NO is oxidized in aerobic systems and the toxicity of these resulting strong oxidants [9]. On the other hand, reduced nitrogen oxides (relative to NO) such as hydroxylamine (NH_2_OH), nitroxyl (HNO), and ammonia (NH_3_) have received much less attention [10] although there are several reports that suggest they can be generated endogenously [11]. These compounds were studied in the past with regard to their biological activity/toxicity [12]. Among the reduced forms, nitroxyl (HNO) is the least understood but is rapidly emerging as a novel entity with distinct pharmacology and therapeutic advantages over the common nitrogen oxide species [13].

RETRACTED

## 2. Nitroxyl (HNO)

In 1896, the Italian scientist Angeli published the synthesis of the inorganic salt Na_2_N_2_O_3_ [14] and several years later proposed its aqueous degradation produced nitrite and NOH [15]. The decomposition mechanism of Angeli's salt (AS) was revised more than a century later; and the products are now well established to be nitrite and the more stable HNO isomer [16]. Nitroxyl (variously called nitrosyl hydride, hydrogen oxonitrate (IUPAC), nitroso hydrogen, or monomeric hyponitrous acid) is a compound related to NO by 1-electron reduction and protonation [17]. Nitroxyl has a very unique biological profile which is distinct from that of its redox cousin NO [18]. Nitroxyl is growing as a potential therapeutic agent for congestive heart failure (CHF) as will be discussed [19, 20]. Nitroxyl appears to be a simple triatomic species, but it possesses novel and atypical chemistry. Prior to 2002, the biologically relevant form of HNO was thought to be the deprotonated anion, NO^−^, since the generally accepted p*K*_*a*_ for HNO was 4.7 [21]. However, recent studies revised the p*K*_*a*_ significantly upward, to approximately 11.4, making HNO the exclusive species present at biological pH [22–24]. In addition, the different spin states of the two species HNO/NO^−^ complicate the acid-base relationship between them [17]. NO^−^, which is isoelectric to molecular oxygen O_2_, has a triplet ground state and a singlet lowest excited state, while the HNO ground state is a singlet. Thus, the HNO acid-base equilibrium species possess different electronic spin states (i.e., protonation-deprotonation is spin forbidden) and it is expected that the rates of protonation and deprotonation will be extremely slow compared to normal acid-base reactions [24]. This spin forbidden transformation supports the idea that the observed biological activity is attributed to the protonated form HNO [17, 24].

RETRACTED

Another complex feature of HNO that complicates the study of the production, detection, and its chemistry is the high reactivity. Chemically, HNO is a highly reactive electrophile that spontaneously dimerizes to give hyponitrous acid, which dehydrates to give nitrous oxide (N_2_O) and water (see (1)) [17, 25, 26]. Detection of N_2_O as an end product may serve as a marker for the involvement or at least the presence of HNO in biological systems [27]. This reaction has been studied both theoretically and experimentally and several rate constant values have been offered with the accepted value, determined by flash photolysis techniques at room temperature, being *k* = 8 × 10^6^ M^−1^ s^−1^ [24]:

(1) $$\begin{array}{c} \text{HNO}+\text{HNO}⟶\text{HON=NOH}⟶N_{2}O+H_{2}O \end{array}$$

Thus, unlike most commonly used nitrogen oxides, HNO cannot be stored or concentrated and is typically studied using donor species that release HNO as a decomposition product.

## 3. Nitroxyl Donors

### 3.1. Angeli's Salt

As mentioned, Angeli's salt (AS) or sodium trioxodinitrate (Na_2_N_2_O_3_) is the most common HNO donor currently used. Angeli's salt releases HNO with a half-life of approximately 2-3 min at physiological pH and temperature. Nitroxyl release from this compound is observed between pH values 4 and 8 [28], through a first-order process, and the generally accepted mechanism involves protonation of the dianion followed by tautomerization and heterolytic cleavage of the N–N bond to produce HNO and nitrite (Scheme 2) [16]. ^15^N-labelling confirms that HNO originates solely from the nitroso group while the nitrite's origin is from the nitro group [29].

Interestingly, when the pH drops below 4, the rate of AS decomposition significantly accelerates, and NO becomes the only nitrogen-containing end product. At higher pH (pH > 8), the decomposition rate decreases. Such a decay profile is extremely useful for practical purposes, as stock solutions of AS are relatively stable at high pH, while the release profile is pH insensitive near physiological conditions. However, the fact that 1 equivalent of nitrite is coproduced during AS decomposition may disturb the experimental interpretation considering the fact that nitrite has its own physiological profile [16].

### 3.2. Piloty's Acid

*N*-Hydroxysulfenamides (Piloty's acid and its derivatives) are another class of HNO donors that have been examined in detail. Piloty's acid shares some similarities with AS including pH-dependent first-order decomposition. Piloty's acid is stable at low pH and its decomposition rate increases at higher pH (Scheme 3). Significant HNO release occurs at pH values higher than biological conditions, while at physiological pH many of Piloty's acid analogs are oxidized and subsequently release NO, not HNO. This pH restriction has limited the use of these compounds as HNO donors in biological studies [30].

RETRACTED

### 3.3. Cyanamide

Cyanamide, an antialcoholic drug used in Canada, Europe, and Japan, was found to be bioactivated via oxidation by the enzyme catalase leading to an* N*-hydroxycyanamide intermediate. This intermediate species spontaneously decomposes to release cyanide and HNO (Scheme 4), which targets a thiol containing enzyme in the metabolic pathway of ethanol (aldehyde dehydrogenase, ALDH) [31, 32].

The release of cyanide during this reaction has restricted the use of cyanamide and its derivatives in biological settings. However, this drug demonstrates the feasibility of clinical use of HNO donors and the ability to selectively target protein thiols as will be seen later [9].

### 3.4. Diazeniumdiolates as HNO Donors

Diazeniumdiolates (NONOates) which are complexes of secondary amines and NO share the same chemical class as AS but they fragment back to NO under the same conditions in which AS decomposes to HNO [33–35]. In contrast to these NO donors, decomposition in neutral solution of the amine NONOate produced with primary amines (isopropylamine, IPA/NO) results in HNO release, while NO forms only at lower pH values, similar to AS [36]. Dutton et al. [37] showed that the mechanism of HNO formation is similar to that of AS, starting from protonation of N(1), followed by slow tautomerization forming a higher-energy isomer protonated at N(3). This tautomer will be a very minor component of the equilibrium but once formed it will spontaneously and rapidly dissociate to produce HNO and the deprotonated nitrosamine because of the very small barrier to N–N bond cleavage (Scheme 5). The resulting nitrosamine is expected to be unstable and rapidly decompose to the primary alcohol and N_2_ [38].

### 3.5. Acyl Nitroso Compounds

Acyl nitroso compounds were observed as an oxidation product of hydroxyurea (a drug that is used for sickle cell disease), and they rapidly hydrolyze to yield N_2_O as evidence for HNO release. Cycloadducts with conjugated 1,3-dienes and N–O heterodienophiles stabilize the acyl nitroso compounds and then they can undergo retro-Diels Alder reactions to yield the parent acyl nitroso compound that rapidly hydrolyses to yield HNO (Scheme 6) [39].

### 3.6. Acyloxy Nitroso Compounds

A new class of HNO donors, acyloxy nitroso derivatives of cyclohexane, has been developed by King's group [40, 41]. They are easily synthesized from oxidation of cyclohexanone oxime or dihydro-2H-pyran-4(3H)-one oxime by either lead tetraacetate (LTA) [40] or (diacyloxyiodo)benzene [42]. They release HNO upon cleavage of the ester bond (Scheme 7). Modifying the electronic and/or steric properties of the acyl group position changes the rate of ester cleavage and thus HNO release. One of the major benefits of these HNO donors, besides controlling the HNO release rate, is that nitrite is not a product as is the case with AS. Another advantage of these compounds that makes them very useful in biochemical studies is the blue color that is a result of the *n* → *π* ^*∗*^ electronic transition of the N–O bond, allowing biochemical reaction kinetics to be easily monitored [40].

RETRACTED

Changing the substitution in such group of compounds greatly determines their properties. 1-Nitrosocyclohexyl trifluoroacetate decomposes immediately releasing HNO upon addition of water or buffer solution in a manner that resembles Angeli's salt ability to release HNO, while 1-nitrosocyclohexyl pivalate is considerably stable with *t*_1/2_ of 2260 min in a 1 : 1 mixture of MeOH : Tris buffer (50 mM, pH 7.6) and hence it is not considered as a common HNO donor [43].

## 4. Endogenous Production of HNO

Since the discovery of endogenous NO generation, carbon monoxide (CO) [44] and hydrogen sulfide (H_2_S) [45] have also joined the ranks of gaseous/small molecule signaling species. The potency by which HNO elicits many of its pharmacological actions and the apparent selectivity of HNO towards several of its established biological targets suggests that the actions of pharmacologically administered HNO are the result of preexisting signaling pathways which responds to HNO. Some reports even assumed that HNO can serve as the endothelium-derived relaxing and hyperpolarizing factor that might contribute to NO claimed vasorelaxing actions [46]. However, no confirmed evidence exists for HNO endogenous generation and this might be due to the lack of a specific and sensitive trap for HNO that can be applied for biological systems. Numerous* in vitro* chemical studies provide possible chemical pathways for that to occur.

Several reports showed that HNO can be produced by NOS under certain conditions [47–50] especially in the absence of its vital prosthetic group, tetrahydrobiopterin [47, 51], and via the metabolism of the NOS product* N*-hydroxy-l-arginine (NOHA) under oxidative stress [52]. Nitroxyl can be also formed under nitrosative stress (e.g., reaction of NO with hydroxylamine yields HNO) [53] and by thiolysis of* S*-nitrosothiols (RSNO, a well characterized species formed in biological systems as a result of NO generation) [2] following thiol nucleophilic attack on the SNO sulfur (see (2)) [11, 26]. Hence,

(2) $$\begin{array}{c} \text{RSNO}+\text{RSH}⟶\text{RSSR}+\text{HNO} \end{array}$$

The direct reduction reactions of NO by mitochondrial cytochrome* c* [54], xanthine oxidase [55], Cu- and Mn-containing superoxide dismutase (CuMnSOD) [56], and ubiquinol [57] are among other reactions reported to generate HNO.

RETRACTED

Oxidation of NH_2_OH can serve as an alternative source for HNO production. The generation of high-valent iron-oxo complexes from the reaction of ferric hemes (usually peroxidases or catalases) with hydrogen peroxide can oxidize NH_2_OH to HNO (Scheme 8) [27, 58].

## 5. Biological Chemistry of HNO

Nitroxyl is a highly reactive electrophile, and the literature on the chemistry of HNO includes multiple examples of reactivity with nucleophiles, oxidants, and metalloproteins [59]. Bartberger et al. [22] used quantum mechanical calculations to predict that HNO reacts somewhat selectively with nucleophiles. Theoretical examination predicts that HNO will not significantly hydrate or react with alcohols; however, it appears to be very reactive towards thiols, with the reaction with amines intermediate between water/alcohol and thiols. These reactions are different from reactions of NO with those nucleophiles.  Table 1 summarizes the main possible reactions of NO and HNO with biological reactants.

### 5.1. Reaction with Thiols

To date, thiols appear to be a major site of HNO biochemical reactivity. Doyle et al. [59] produced one of the earliest reports of thiol reactivity with HNO showing a 98% yield of disulfide and NH_2_OH as the final products of the reaction of HNO with thiophenol in 40% aqueous acetonitrile (see (3)). This yield suggested that the rate of this reaction significantly exceeds the rate of HNO dimerization (see (1)) [17]:

(3) 2C6H5SH+HN2O3−⟶C6H5SSC6H5+NH2OH+NO2−

Further thiol reactivity was reported with other biologically relevant thiols such as reduced glutathione (GSH) [26],* N*-acetyl-l-cysteine (NAC) [60], and dithiothreitol (DTT) [61]. The mechanism for this reaction was suggested to include an attack of the nucleophilic sulfur on the electrophilic nitrogen atom of HNO leading to the formation of an* N*-hydroxysulfenamide intermediate. The* N*-hydroxysulfenamide intermediate can further react with excess thiol (or a vicinal protein thiol) to give the corresponding disulfide and hydroxylamine (Scheme 9) [59] or rearrange to sulfinamide in a competing reaction (Scheme 9) [26].

Significantly, disulfide formation is considered to be biologically reversible because disulfides are easily regenerated while the generation of the sulfinamide apparently represents an irreversible thiol modification [62]. The rate of some of these reactions was also investigated and for GSH the rate constant was found to be *k* = 2 × 10^6^ M^−1^ s^−1^ [25]. The HNO-thiol reaction was also reported to be condition dependent (under high thiols concentration the disulfide is the main product while under low reduced thiol concentration the* N*-hydroxysulfenamide intermediate rearranged to the sulfinamide) [17, 26, 60].

RETRACTED

This reactivity with thiols indicates that protein sulfhydryl groups may be a major target for HNO. Shen and English characterized a similar type of chemistry using electron spray ionization mass spectrometry (ESI-MS) upon the reaction of AS with thiol proteins, such as bovine serum albumin (BSA), glyceraldehydes-3-phosphate dehydrogenase (GAPDH), and human brain calbindin (HCalB). They used MS characters of whole proteins and their digests to demonstrate the ability of HNO to induce disulfide bond formation when these reactions were done in the presence of excess cysteine, while, with no excess thiols, the sulfhydryl group present in these proteins was converted mainly to sulfonamide [63]. Other reports suggest the ability of these sulfinamides to be hydrolyzed to sulfinic acids (SO_2_H) [64, 65]. The rate of the reaction between HNO and thiol proteins appears to be faster than that with small thiols, as the cysteine in BSA reacts with a rate constant of *k* = 6 × 10^6^ M^−1^ s^−1^. It can be estimated that GAPDH, with a low p*K*_*a*_ thiol, reacts at a rate >10^9^ M^−1^ s^−1^. Thus, thiol p*K*_*a*_ and hydrophobicity of the thiol environment influence the reactivity [66].

Hoffman and coworkers used a tandem mass spectrometric analysis including MS/MS with collision induced dissociation (CID) and electron capture dissociation to identify the sulfinamide modification introduced by AS to thiol proteins. These studies revealed a characteristic neutral loss of HS(O)NH_2_ fragment (65 Da) that is liberated from the modified cysteine upon CID monitored by mass spectrometry. Upon storage, partial conversion of the sulfinamide to sulfinic acid was observed, leading to neutral losses of 65 and 66 Da (HS(O)OH) [64].

These experimental data are supported by theoretical calculations for the free energies involved in the reaction of HNO with 5 different thiols. The reaction was found to be dependent on the loss of the S–H proton, a requirement for S–N bond formation. These findings were consistent with proteins whose environment favors the existence of thiolate anions being selectively inhibited by HNO. This work also showed that protonation of the HNO oxygen atom may also be required before or during the rate limiting step. The authors strongly suggest that the competition between the two possible pathways would be kinetically controlled. Additionally, the calculated values of Δ*G* indicate that the preferred reaction pathway depends upon the hydrophobicity of the environment, the availability of a local base, and the identity of the thiol substituent. In a hydrophobic environment, the calculated activation barriers strongly indicate that formation of a disulfide is favored, consistent with the ability of GSH to prevent the irreversible inhibition of proteins* in vitro*. The formation of the sulfinamide would be expected to become more favorable if a base was present in the local environment and with stronger electron-withdrawing substituents on the thiol. In solution, a greater competition between the two pathways is predicted, but formation of the disulfide is expected to be favored in most conditions [67].

RETRACTED

### 5.2. Reaction with Metals/Metalloproteins

Another aspect of HNO chemistry important for its biological activity is its ability to react and/or form coordination complexes with metalloproteins, particularly iron heme proteins [68]. Nitroxyl reacts with oxidized metals to form reductive nitrosylation products in a single step reaction; this reaction was originally observed upon exposure of metmyoglobin (metMb) or methemoglobin (metHb) to AS (see (4)) [59, 69]:

(4) $$\begin{array}{c} \text{Fe}\left(\;\text{III}\;\right)+\text{HNO}⟶\text{Fe}\left(\;\text{II}\;\right)\text{NO}+H^{+} \end{array}$$

Other ferric proteins including cytochromes, peroxidases [69], and catalases [70] also undergo reductive nitrosylation by HNO, indicating lack of specificity toward nitrogen (histidine), sulfur (cysteine or methionine), and oxygen (tyrosine) as the protein part that binds to iron next to the HNO binding site. The protein environment around this site may have significant impact on the kinetics of reductive nitrosylation [17].

The suggested mechanism for this reaction is either an inner sphere mechanism, whereby direct coordination of HNO to the metal center occurs followed by electron transfer and deprotonation, or via an outer sphere mechanism involving initial electron transfer to the metal center followed by coordination of NO to the reduced metal center. The existence of an outer sphere process is evident in the reaction of HNO with ferricytochrome c, which only produces the ferrous species and NO [59]. The rate constant of these reactions was estimated for the reaction of synthetic ferric porphyrin with AS to be *k* = 3 × 10^5^ M^−1^ s^−1^ (comparable to that with metMb *k* = 8 × 10^5^ M^−1^ s^−1^) [71].

Nitroxyl also reacts with oxyhemes (e.g., oxymyoglobin, MbO_2_, and Fe(II)O_2_) converting two MbO_2_ to two metMb (Fe(III)) with a rate constant of 10^7^. A two-step reaction was proposed with the intermediacy of NO and formation of peroxide (see (5)-(6)); the formed peroxide can react to generate a ferryl-*p*-cation radical. As this reaction has not been confirmed, there is a possibility that HNO is reduced to H_2_NO rather than being oxidized to NO with rapid dissociation of the resulting Fe(III)O_2_ complex (see (7)-(8)) [17, 66]:

(5) FeIIO2+HNO⟶FeIII+NO+HO2−

(6) FeIIO2+NO⟶FeIII+NO3−

(7) FeIIO2+HNO⟶FeIII+H2NO+O2

(8) FeIIO2+H2NO⟶FeIII+NH2OH+O2

Other metalloproteins also have been reported to react with HNO. CuZnSOD reacts with HNO to yield NO [69], while reaction with MnSOD results in a Mn–NO complex [72].

RETRACTED

### 5.3. Reaction with Phosphines

Previous reports showed reactions of organic phosphines with various nitroso compounds. C-Nitroso and S-nitroso compounds react with triphenylphosphine (TPP) and similar triarylphosphines to form phosphine oxides and aza-ylides [73–75]. Reisz et al. reported a similar type of phosphine reactivity toward HNO (viewed as a simplified nitroso compound) (Scheme 10) [76].

The proposed mechanism for this reaction was P addition to N or O of the nitroso group forming a three-membered ring intermediate, which upon reaction with additional equivalent of phosphine would give the corresponding aza-ylide and phosphine oxide.

This work also showed that, in the presence of an electrophilic ester, properly positioned on the phosphine, the aza-ylide undergoes Staudinger ligation to yield an amide with the nitrogen atom derived from HNO (Scheme 11) [76].

### 5.4. Other HNO Reactions

Nitroxyl reacts with O_2_ to form an RNS (reactive nitrogen species) which does not appear to be peroxynitrite (ONOO^−^) but has some similar chemistry [77, 78]. This species is a strong 2e^−^ oxidant and hydroxylating agent and is cytotoxic at low millimolar concentration and causes DNA strand breaks [53, 77]. The rate of this autoxidation of HNO is relatively slow (*k* = 1000 M^−1^s^−1^) compared to the rate of HNO reactivity with other biological reactants like GSH, and the lower concentration of O_2_ relative to the other biomolecules severely limits the formation of this species* in vitro* and consequently limits the oxidative damage due to the exposure to HNO* in vivo *[17].

Other RNS could be formed indirectly from HNO, after its oxidation to NO with superoxide dismutase (SOD) [66]. N_2_O_2_^−^ also can be formed from the reaction of HNO and NO at a rate constant of 5 × 10^6^ M^−1^s^−1^ [66]. Nitroxyl can react with other nucleophilic nitrogen oxides such as hydroxylamine (see (9)) and nitrite (reverse of Scheme 2):

(9) $$\begin{array}{c} {NH}_{2}OH+HNO⟶N_{2}+2H_{2}O \end{array}$$

Nitroxyl reduction to NH_2_OH can easily occur under physiological conditions. This was confirmed by calculation of the reduction potential for the HNO, 2H^+^/NH_2_OH couple at pH 7 to be 0.3 V [24]. It was proposed that NH_2_OH might be the product of HNO oxidation of NADPH by two electrons to NADP^+^ though this has not been confirmed [79].

RETRACTED

## 6. Detection of HNO

Several methods implicate the presence or fleeting existence of HNO. As mentioned, the detection of N_2_O has been used as evidence for HNO generation since HNO spontaneously dimerizes to hyponitrous acid (H_2_N_2_O_2_) that then decomposes to N_2_O and water (see (1)). N_2_O is usually detected by gas chromatography-mass spectrometry (GC-MS). However, this cannot be applied to biological samples as an absolute proof of HNO intermediacy since N_2_O can be generated in ways not involving free HNO [80]. Moreover, N_2_O formation is second order in HNO and requires fairly high concentrations for this reaction to be significant.

As discussed earlier, HNO reacts readily with thiols. In fact, Pino and Feelisch [81] used thiol reactivity as a means of trapping HNO and distinguishing its actions from those of NO. Furthermore, the identification of the HNO based thiol modification could serve as a useful method for HNO detection. Donzelli et al. [27] used HPLC techniques to identify both the sulfinamide [GS(O)NH_2_] and the oxidized glutathione (GSSG) as evidence of GSH exposure to AS.

Transition metals can also be used to trap HNO, with the highest applicability of metMb or synthetic analogs and trapping to produce EPR active species [82, 83]. Other methods involved the oxidation of HNO to NO using ferricyanide and then detecting the formed NO with chemiluminescence or electrochemical analysis techniques [84].

Shoeman and Nagasawa [85] reported that nitrosobenzene could trap HNO to give cupferron (Scheme 12), a species that complexes copper forming a colored complex. However, this has not yet been exploited for the detection of HNO in a biological system, and the efficiency of this trap has not yet been determined.

The use of water soluble phosphines represents a powerful way to trap HNO in biological samples by tracking the aza-ylide (Scheme 10) that is formed upon the reaction of HNO with phosphines using simple ^31^P NMR techniques [76].

HPLC and colorimetric methods were developed by Reisz et al. to quantify HNO release from donor compounds using phosphine derivatives. Ligation of HNO using carbamate containing phosphine derivatives yielded HNO derived urea (Scheme 13) and the corresponding phenol. Starting with a nitro derivatized phosphine trap yielded* p*-nitrophenol that can be monitored calorimetrically [86].

RETRACTED

HNO reaction with GSH was also used for HNO detection. HNO was trapped by GSH followed by labeling of GSH with the fluorogenic agent, naphthalene-2,3-dicarboxaldehyde (NDA), and subsequent quantitation by fluorescence difference [87].

A prefluorescent probe, 4-((9-acridinecarbonyl)amino)-2,2,6,6-tetramethylpiperidin-1-oxyl (TEMPO-9-AC), has been used to detect HNO in aqueous solution and to differentiate it from nitric oxide (NO). TEMPO-9-AC reacts with HNO via net hydrogen abstraction to produce the highly fluorescent TEMPO-9-AC-H and NO. The utility of TEMPO-9-AC as a probe for HNO has been shown using the common HNO donors Angeli's salt and Piloty's acid (PA) along with a recently reported HNO donor, 2-bromo-PA [88].

Recently, a near-infrared fluorescent turn-on sensor for the detection of nitroxyl (HNO), using a copper-based probe, CuDHX1, was recently developed for selective quantitation of HNO in biological samples. The probe contains a dihydroxanthene (DHX) fluorophore and a cyclam derivative as a Cu(II) binding site. Upon reaction with HNO, CuDHX1 displays fivefold fluorescence turn-on in cuvettes and is selective for HNO over thiols and reactive nitrogen and oxygen species [89].

Clearly, the development of sensitive, specific, and biologically compatible traps/detectors for HNO is essential in determining whether HNO is physiologically relevant. Moreover, such methodology will be valuable for future investigations distinguishing the specific actions of HNO from those of other nitrogen oxides.

## 7. Biological Activity of HNO

Endogenous HNO generation remains uncertain in mammalian cells. Therefore, the question of whether HNO is a natural signaling/effect or species remains open. However, numerous studies indicate that exogenous HNO administration results in interesting, novel, and potentially important pharmacology and toxicology [62].

### 7.1. HNO and Antialcoholism

The first report of HNO serving as a drug was from the Nagasawa research group who were examining the action of the antialcoholic drug cyanamide [31, 32, 90]. The utility of this drug lies in its ability to inhibit ALDH, an enzyme involved in the metabolism of ethanol to acetate. Cyanamide has no inherent activity and must be oxidatively bioactivated to elicit enzyme inhibition. Oxidation of cyanamide by catalase/H_2_O_2_ generates an* N*-hydroxy intermediate that decomposes to HNO and cyanide as shown in Scheme 4. Inhibition of ALDH was proposed to occur via reaction of HNO with the active site cysteine thiolate of the enzyme. This finding was among the first indications that HNO was thiophilic and could alter the actions of thiol proteins.

RETRACTED

### 7.2. HNO and Vascular Function

Similar to NO, HNO acts as a potent vasorelaxant [91]. Angeli's salt elicits vasorelaxation in isolated large conduit [92, 93], small resistance arteries [94], and intact coronary [95] and pulmonary [96] vascular beds, in both rabbits [97] and dogs [98, 99]. Acyloxy nitroso compounds also caused dilatation in thoracic aorta isolated from Sprague-Dawley rats in a dose-dependent manner [43]. Paolocci et al. showed that HNO shows selectivity being a venodilator in contrast with NO donors that equally dilate both arteries and veins. In addition, they showed HNO's ability to decrease mean arterial blood pressure [99]. Recently, HNO is introduced as a vasodilator for humans that is not susceptible to tolerance [100].

Because NO elicits vasodilation via activation of sGC [101], it is possible that HNO was being converted to NO in these experiments. Such conversion seemed especially likely because HNO itself has been reported to be incapable of activating sGC [102], although these studies were performed under high thiol conditions that probably scavenged HNO. Like NO, vasorelaxant responses to HNO are accompanied by an increase in cGMP [103] and are impaired by the sGC inhibitor, 1*H*-[1,2,4]oxadiazolo[4,3-a]quinoxaline-1-one (ODQ) [92, 95, 103], indicating that HNO targets sGC. Whether HNO itself directly activates sGC or first requires oxidation to NO, or if the preference of HNO for Fe(III) versus Fe(II) targets its actions to the oxidized, NO-insensitive sGC isoform, which predominates in disease, remains to be determined [104]. Zeller et al. [105] support the idea of HNO being oxidized first to NO by the enzyme SOD before activating sGC, but further investigations are required.

Nitroxyl, but not NO, increases the plasma level of the vasodilatory neuropeptide calcitonin gene related peptide (CGRP) [98, 99]. Calcitonin gene related peptide stimulates endothelial NO release, increases vascular smooth muscle cAMP, and activates K^+^ channels to elicit vasodilatation [25, 106]. However, the use of antagonist, CGRP, does not prevent* in vivo* vasodilatation of HNO, suggesting that CGRP may not contribute to HNO's actions [99]. Although CGRP seems to contribute to AS mediated coronary vasodilation* ex vivo* [95], it remains unclear how HNO stimulates* in vivo* CGRP release and whether CGRP plays a similar role in other vascular beds. Recent report suggested that HNO endogenously produced via the reaction of NO with H_2_S can form a disulfide bond in the sensory chemoreceptor channel TRPA1 resulting in sustained calcium influx that causes release of CGRP [107].

RETRACTED

HNO also targets K^+^ channels to modulate vascular function. Multiple studies show that both K_v_ and K_ATP_ channels were affected in HNO-mediated vascular and nonvascular smooth muscle relaxation [46, 94]. By contrast, NO only activates K_Ca_ channels in this preparation [108]. Nitroxyl activation of K^+^ channels may be direct or cGMP-dependent and HNO-thiol interactions could enable direct modulation of K_v_ and K_ATP_ channels independently of cGMP [94].

The vasodilatory capacity of HNO donors and their ability to target signaling pathways distinct from NO might offer therapeutic advantages over traditional nitrovasodilators. Several reports demonstrated that, unlike organic nitrates such as glyceryl trinitrate (GTN), AS does not develop tolerance after either acute or chronic use [100, 103]. Given that AS inhibits the thiol protein ALDH-2 [9], which has an important role in GTN biotransformation to NO [109], cross-tolerance between AS and GTN is not likely to happen which may be of interest [103]. Nitroxyl donors could have novel utility as vasodilators, alone or in conjunction with conventional nitrovasodilators, in the treatment of vascular disorders such as angina and heart failure [13].

### 7.3. HNO and Myocardial Function

Originally, the pharmacological utility of HNO in the cardiovascular system was considered limited to vasodilation. More recently, HNO donors have been shown to be capable of profoundly affecting myocardial contractility [18].

Nitroxyl has been shown to have positive inotropic (force of muscle contraction) and lusitropic (relaxation of cardiac muscle) properties; both properties contribute to increased cardiac output in both normal and failing canine hearts. In this study, Paolocci et al. utilized a pressure-volume relationship approach to examine primary effects of HNO on the heart from changes in vascular loading conditions and demonstrated for the first time that AS was capable of increasing the inotropic status of the heart while fastening ventricular relaxation and unloading of the heart [99].

Nitroxyl-mediated inotropy was not mimicked by an NO donor and is prevented by the HNO scavenger NAC indicating a direct HNO effect. In dogs with tachypacing- induced congestive heart failure (CHF), HNO improved both contractility and relaxation to an extent similar to that found for control dogs [98]. Nitroxyl inotropy was not dependent on beta-adrenergic pathways and was additive to beta-adrenergic agonists in enforcing myocardial contractility. Positive inotropy, unloading cardiac action, and peripheral vasodilation are all desirable outcomes in CHF subjects. Current CHF cases are usually treated via beta-agonists or phosphodiesterase inhibitors, giving inotropic support to the heart, and through nitrosovasodilators, to unload the heart. That HNO donors provide both effects together is a unique advantage.

RETRACTED

Tocchetti et al. [110] and others [19] have explained the increased myocardial contractility by showing that HNO elicits the prompt release of Ca^2+^ from the sarcoplasmic reticulum (SR) in both cardiac and skeletal muscle via activation of ryanodine receptors (RyR2) and skeletal Ca^2+^ release channels (RyR1). These effects appear to occur through modifications of certain thiol residues in these receptors. In both cases, the effects were reversible upon the addition of a sulfhydryl reducing agent, DTT.

Froehlich et al. [111] suggested that HNO donated by AS can also activate Ca^2+^ uptake by the cardiac SR Ca^2+^ pump (SERCA2a) by targeting the thiols in phospholamban (PLN, a regulatory protein that controls SERCA2a). They concluded that HNO produces a disulfide bond that alters the conformation of PLN, relieving inhibition of the Ca^2+^ pump. This increase in uptake keeps the net diastolic Ca^2+^ low.

In addition to these changes in Ca^2+^ cycling, HNO also acts as a cardiac Ca^2+^ sensitizer, enhancing myofilament responsiveness to Ca^2+^ and augmenting maximal force of myocardial contractility. This effect is likely to be due to modulation of myofilament proteins that have many reactive thiolate groups and are potential targets of HNO. Altering intracellular redox conditions with DTT prevented HNO-induced augmentation in muscle force development, consistent with the idea of HNO affinity for strategically located thiols [112].

These combined mechanisms suggesting the orchestrated action of HNO with cardiac myofilaments and SR to enhance inotropy and lusitropy at potentially lower energetic cost make HNO an attractive candidate for CHF cases.

### 7.4. HNO and Ischemia Reperfusion Injury

Nitroxyl also elicits effects in ischemia reperfusion (IR) injury. Ischemia reperfusion injury occurs when tissue is deprived of adequate blood flow for a period of time causing hypoxia, which is the ischemic event, and other effects. Reperfusion of oxygenated blood causes the injury and results in necrosis of the tissue. Ischemia reperfusion injury can be alleviated by preconditioning the tissue, which involves brief occlusions of the vasculature prior to the actual cessation of blood flow. Administration of AS to ischemic myocardium was found to be detrimental, as opposed to the beneficial effects exerted by equieffective doses of NO donors [97]. No clear-cut mechanisms for the HNO exacerbation of injury were identified, though a possible explanation may be the ability of HNO to induce neutrophil accumulation [9]. Pagliaro and coworkers later showed that HNO is capable of inducing early preconditioning-like effects in isolated rat hearts to an extent even greater than that induced by NO donor [113]. Again this protective signaling cascade is not clear, with Shiva and coworkers suggesting that mitochondrial thiols are possible HNO targets [114]. Additionally, CGRP may mediate a part of HNO ability to induce protection, as CGRP has been reported to be protective in this context [115].

RETRACTED

Furthermore, the distinct role of HNO in cardiovascular system made it a very promising strategy in treatment of cardiomyopathy associated with various diseases such as diabetes. The HNO donor 1-nitrosocyclohexylacetate (1-NCA) was proven to limit cardiomyocyte hypertrophy and LV diastolic dysfunction in a mouse model of diabetes* in vivo* [116].

### 7.5. HNO and Platelet Aggregation

Treatment of platelets with micromolar concentrations of AS leads to inhibition of platelet aggregation in both time- and dose-dependent fashion [117]. Hoffman et al. [64] identified the ability of HNO to induce modifications in 21 proteins within human platelets, with 10 of those proteins showing dose-dependent modification. The function of these proteins ranges from metabolism and cytoskeletal rearrangement to signal transduction.

### 7.6. HNO and Anticancer Activity

In early 2008, Brooks reported the anticancer activity of HNO by demonstrating the ability of HNO to suppress the proliferation of both estrogen receptor- (ER-) positive and ER-negative human breast cancer cell lines, in a dose-dependent manner. This inhibition was accompanied by a significant decrease in the blood vessel density in HNO-treated tumors. Both* in vitro* and* in vivo* models of breast cancer were used to evaluate AS. One explanation for this activity is the ability of HNO to inhibit the thiol protein glyceraldehydes-3-phosphate dehydrogenase (GAPDH) blocking the glycolytic cycle inside the malignant cell and leading to a cascade of signaling mechanisms resulting in the inhibition of angiogenesis [118]. Nitroxyl inhibition of GAPDH was previously reported leading to inhibition of glycolysis in yeast cells [119, 120].

In the next year, Froehlich also reported the ability of HNO to suppress the growth of both hormone dependent and independent cancers such as prostate, breast, pancreatic, and lung cancer that overexpress a protein called MAT-8 protein (mammary tumor 8 kDa protein) [121, 122]. MAT-8 is member of the family of FXYD regulatory proteins; it inhibits the plasma membrane Na^+^/K^+^ pump causing collapse of the transmembrane Na^+^ gradient [123], affecting cellular Ca^2+^ levels that protect tumor cells from apoptosis [124]. Froehlich demonstrated that HNO inhibited the MAT-8 protein via disulfide bond formation between transmembrane cysteine residues, relieving the Na^+^/K^+^ pump inhibition and triggering endoplasmic reticulum stress, rendering the cell susceptible to apoptosis and destruction [125].

RETRACTED

### 7.7. HNO and Antioxidant Activity

Chemistry predicts that HNO can serve as an antioxidant, with its relatively weak H–N bond strength of ~50 Kcal/mol, making it a good hydrogen atom donor, with the ability to quench reactive radical species [28]. HNO capably inhibits lipid peroxidation in both yeast and* in vitro* model systems [126]. Nitroxyl inhibits free radical lipid oxidation by interacting with the initiating agent, lipid radical or lipid peroxy radical, thus terminating the radical chain chemistry (see (10)–(13)). Oxidation of HNO gives NO that can also quench radical intermediates [9]:

(10) L–H+In∙⟶L∙+In–H L=lipid, In⁡=free  radical  initiator

(11) In∙+HNO⟶In–H+NO∙

(12) L∙+HNO⟶L–H+NO∙

(13) LOO∙+HNO⟶LOO–H+NO∙

### 7.8. HNO and Central Nervous System (CNS)

Nitroxyl also interacts with the thiol residues on the* N*-methyl-d-aspartate (NMDA) receptor that plays a vital role in neuronal communication and synaptic function in the CNS [127]. Since overstimulation of the NMDA receptor has been implicated in the excitotoxicity associated with glutamate, the physiological outcome of this HNO action affords protection against glutamate-based excitotoxicity. In contrast, Colton and coworkers [128] reported that HNO was also capable of blocking glycine-dependent desensitization of the NMDA receptor resulting in net sensitization of the receptor. The suggestion was made that the divergent outcomes of these studies are at least in part a function of O_2_ depletion upon long term use of AS, which consumes O_2_ during decomposition. Thus, careful attention needs to be paid to experimental conditions, particularly with regard to O_2_ and metal content. However, both studies indicate that HNO can modify the activity of the NMDA receptor, in either a positive or a negative fashion, depending on the oxygen tension of the system [9].

### 7.9. HNO and Other Thiols

In addition to the thiol proteins mentioned in the previous sections, HNO is a potent inhibitor of some cysteine proteases like papain [129] and cathepsin P [130, 131]. It also inhibits the metal responsive yeast transcription factor Ace1 [132] and depletes intracellular GSH levels [53].

### 7.10. HNO Toxicity

Cyanamide is the only clinically approved drug that functions exclusively through release of HNO. The therapeutic use of cyanamide induces little inherent toxicity at prescribed doses indicating that administration of HNO donors is not inherently toxic.

RETRACTED

However, some* in vitro* experiments showed some toxicity associated with the use of AS in very high concentrations compared to those used for biological studies. AS was found to significantly reduce cellular viability, due to severe depletion of cellular GSH levels. Nitroxyl can also induce double-stranded DNA breaks. The cytotoxicity of Angeli's salt was substantially diminished under hypoxic conditions, indicating a role for O_2_ in the toxicity of HNO. These observations were observed at 1–3 mM AS, which significantly exceeds the concentrations of AS utilized in pharmacological applications. The effects observed with cultured cells may not be applicable to* in vivo* systems with intact redox buffering capacity [53].

High concentrations of HNO have been proposed to be responsible for the neurotoxicity observed following administration of AS to rats via intranigral infusion. The effects were both acute and progressive (occurring after the dissipation of HNO). The acute phase was attributed to direct interactions of HNO with cellular components while the delayed phase may be a result of excitotoxicity [133]. Intrathecal administration of Angeli's salt to the lumbar spinal cord of rats resulted in motor neuron injury without effect on sensory neurons [134].

Nitroxyl shows some interactions with mitochondria as a redox active species, though these interactions were not reported to be toxic, and no pharmacological utility was reported also [9]. Inhibition of GAPDH by HNO inhibits cellular glycolysis [119].

In summary, HNO seems to hold very promising therapeutic potential for cardiovascular diseases (especially CHF) due to its activity profile on the heart and vasculature. Enhancement of intracellular Ca^2+^ cycling and myofilament Ca^2+^ sensitization appear to be unique, in addition to vasodilation and reduction in cardiac load. HNO also provides a promising strategy in fighting cancer due to its ability to inhibit GAPDH. Moreover, the bioactivity of HNO appears distinct compared to NO, making biological targeting by HNO localized and specific facilitating the use of HNO as a novel therapeutic agent.

## Figures and Tables

**Scheme 1:** Enzymatic production of NO from l-arginine.

**Scheme 2:** Nitroxyl release from AS.

**Scheme 3:** Nitroxyl release from Piloty's acid.

**Scheme 4:** Nitroxyl release from cyanamide.

**Scheme 5:** Nitroxyl release from IPA/NO.

**Scheme 6:** Nitroxyl release from acyl nitroso compounds.

**Scheme 7:** Nitroxyl release from acyloxy nitroso compounds.

**Scheme 8:** Oxidation of hydroxylamine to HNO by high-valent iron-oxo complexes.

RETRACTED

**Scheme 9:** Reaction of HNO with thiols.

**Scheme 10:** Reaction of HNO with triphenylphosphine.

**Scheme 11:** Staudinger ligation of HNO with triarylphosphines.

**Scheme 12:** Reaction of AS with nitrosobenzene.

**Scheme 13:** Ligation of AS with arylphosphines producing phenols that can be monitored calorimetrically.

**Table 1:** Comparison of NO and HNO reactivity with biological reactants [28].

Biological reactant	NO	HNO
NO	No reaction	Forms N_2_O_2_^−^/HN_2_O_2_ unknown chemistry
HNO	Forms N_2_O_2_^−^/HN_2_O_2_ unknown chemistry	Dimerization and decomposition to N_2_O
O_2_	Autoxidation leading to nitrosative species, that is, NO_2_ and N_2_O_3_	Forms a potent 2e^−^ oxidant that is not ONOO^−^
RSH/RS−	No direct reaction	Forms sulfinamide or disulfide + hydroxylamine
Fe(II) heme	Very stable Fe(II)-NO	Forms coordination complex
Fe(III) heme	Forms unstable electrophilic nitrosyl, first step in reductive nitrosylation	Very stable Fe(II)-NO except sGC
Cu^2+^	No reaction	Reduces Cu^2+^ to Cu^+^ yielding NO
Lipid radical	Yields lipid-NO	Yields lipid-H + NO
